The article "Deep Learning Algorithm for COVID-19 Classification Using Chest X-Ray Images" was published in 2021. Journal: Comput Math Methods Med.

# Deep Learning Algorithm for COVID-19 Classification Using Chest X-Ray Images

**DOI:** 10.1155/2021/9269173

**Published:** 2021-11-09

**Authors:** Sharmila V J, Jemi Florinabel D

**Affiliations:** ^1^Loyola-ICAM College of Engineering and Technology, Loyola Campus, Nungambakkam, Chennai 600034, Tamil Nadu, India; ^2^Dr. Sivanthi Aditanar College of Engineering, Tuticorin District, Thiruchendur 628215, Tamil Nadu, India

## Abstract

Early diagnosis of the harmful severe acute respiratory syndrome coronavirus 2 (SARS-CoV-2), along with clinical expertise, allows governments to break the transition chain and flatten the epidemic curve. Although reverse transcription-polymerase chain reaction (RT-PCR) offers quick results, chest X-ray (CXR) imaging is a more reliable method for disease classification and assessment. The rapid spread of the coronavirus disease 2019 (COVID-19) has triggered extensive research towards developing a COVID-19 detection toolkit. Recent studies have confirmed that the deep learning-based approach, such as convolutional neural networks (CNNs), provides an optimized solution for COVID-19 classification; however, they require substantial training data for learning features. Gathering this training data in a short period has been challenging during the pandemic. Therefore, this study proposes a new model of CNN and deep convolutional generative adversarial networks (DCGANs) that classify CXR images into normal, pneumonia, and COVID-19. The proposed model contains eight convolutional layers, four max-pooling layers, and two fully connected layers, which provide better results than the existing pretrained methods (AlexNet and GoogLeNet). DCGAN performs two tasks: (1) generating synthetic/fake images to overcome the challenges of an imbalanced dataset and (2) extracting deep features of all images in the dataset. In addition, it enlarges the dataset and represents the characteristics of diversity to provide a good generalization effect. In the experimental analysis, we used four distinct publicly accessible datasets of chest X-ray images (COVID-19 X-ray, COVID Chest X-ray, COVID-19 Radiography, and CoronaHack-Chest X-Ray) to train and test the proposed CNN and the existing pretrained methods. Thereafter, the proposed CNN method was trained with the four datasets based on the DCGAN synthetic images, resulting in higher accuracy (94.8%, 96.6%, 98.5%, and 98.6%) than the existing pretrained models. The overall results suggest that the proposed DCGAN-CNN approach is a promising solution for efficient COVID-19 diagnosis.

## 1. Introduction

The coronavirus disease 2019 (COVID-19) pandemic was caused by severe acute respiratory syndrome coronavirus 2 (SARS-CoV-2). The consequences of this pandemic have caused threats to life among the human race. Although mild and moderately affected COVID-19 patients recovered quickly without any special treatment, numerous studies have confirmed that older people are vulnerable to the severe effects of this disease, particularly those with preexisting medical conditions such as cardiovascular disease, diabetes, chronic respiratory disease, and cancer. Coronaviruses (CoVs) fall under the CoV family of order Nidovirales and are nonsegmented positive-sense RNA viruses. CoVs produce 80-160 nm crown-shaped peplomers with positive polarity of 27-32 kb, along with a high pleomorphic rate and mutation. According to the World Health Organization (WHO), COVID-19 has infected over 222,180,532 people worldwide and killed 4,592,893. As per the records, nearly 198,785,372 patients have been treated for CoV (September 7, 2021) [1]. However, due to its low sensitivity, real-time reverse transcription-polymerase chain reaction (RT-PCR), the recent diagnosis technique, provides negative results for patients with disease symptoms that have been diagnosed by computed tomography (CT) or chest radiography (CXR).

CXR is a simple and relatively inexpensive imaging modality available in many resource-constrained healthcare environments. The visual representations of CXR and CT imaging are represented in Figure 1.

The difference between CXR and CT imaging is expressed in Table 1.

Both procedures can assist clinical expertise in determining better treatment plans for patients. In an article, radiologist Wang et al. [2] mentioned the term “ground glass” to indicate the opacity of a hazy lung. CXR diagnoses this dense opacity that obscures the vessel and bronchial walls quickly. In addition, CXR image-based COVID-19 classification provides reliable results for remote village populations [3]. On the other hand, CT images monitor health conditions [4] to provide the severity and extent of the disease. In this study, we divided the cases into nonemergency (mild or common) and emergency (severe or fatal) cases based on clinical and unique imaging characteristics. Visual functions included vascular enlargement of ground-glass opacity (GGO) lesions and traction bronchiectasis. This analysis assisted in diagnosing the stage and severity of the disease. Using CT images to determine the severity of the disease reflected a lower prevalence of lung and multifocal lesions. Therefore, CT images could not differentiate between other lung infections.

In recent years, deep learning has endorsed an exponential research focus and outperformed many conventional models. Deep learning models [5] can effectively learn the CXR image features and reduce the number of training cycles. It is an efficient learning tool that can solve complex and cognitive problems occurring in COVID-19 diagnosis. However, deep learning approaches, such as convolutional neural networks (CNNs), require an enormous amount of training data and can cause overfitting with small datasets. Numerous studies have confirmed that an enormous amount of data enhances the performance of CNNs. Various pretrained models [6] (LeNet, AlexNet, GoogLeNet, VGG16, VGG19, and Resnet50) are available for training deep learning networks. In addition, many open datasets that provide unbalanced image datasets for training are accessible from online resources such as Kaggle and GitHub. To overcome dataset scarcity, we introduced a generative adversarial network (GAN) to generate synthetic/fake images for training CNN. To evaluate the generative capability of the GAN network, a study [7] experimented with different datasets to obtain the number of datasets required to work on the GAN and found that 50,000 images were sufficient to obtain better results rather than the entire dataset. The GAN performance was tested using two distinct datasets (CelebFaces attributes and large-scale scene understanding). GAN reduces the effort and time required to gather large datasets [8]. It [9] is a deep learning model wherein two neural networks interact in a zero-sum game. In this model, we represented two networks: a generator and a discriminator. The discriminator does not succumb to overfitting, even if a limited training sample is utilized. However, although GAN performs satisfactorily in many areas, it causes severe problems in stabilizing the training process. These shortcomings can be avoided by using a deep convolutional generative adversarial network (DCGAN). In CNN, DCGAN discriminators and generators are designed to achieve a higher performance in image synthesis tasks. The stride and fractional strides of convolution in the discriminator replace the pooling layers, allowing the model to obtain its own upsampling and downsampling in the training process. In addition, during the training phase, poor initialization problems are solved by applying batch normalization to both the generator and discriminator. Therefore, the above improvements in DCGAN alleviate the prevailing instability of training a conventional GAN.

Long short-term memory (LSTM) [10] is one of the most extensively used deep learning approaches as it quickly forecasts COVID-19 cases. LSTM captures the sequence pattern information of the training set using specified features. CNN is a popular deep learning method that extracts noise-free valuable knowledge for model forecasting. Adding enormous layers to a CNN improves its prediction accuracy. The main objective of this study is to aid an accurate COVID-19 classification. Therefore, we proposed a DCGAN-CNN approach for accurate COVID-19 classification without data scarcity. The main contributions of this study are summarized below:

1. The proposed CNN model consists of eight convolutional layers, four max-pooling layers, and two fully connected layers for extracting image features
2. DCGAN is an effective technique for generating large datasets
3. CXR images were utilized for gathering the visual index of COVID-19 diseases
4. By combining DCGAN-CNN, learning models have exhibited versatile performance in COVID-19 classification

The remaining part of this research paper comprises four sections: Section 2 (Related Works) explains the related works of COVID-19 diagnosis models; Section 3 (Proposed Method) elaborates the proposed model DCGAN-CNN; Section 4 (Results and Discussion) represents the experimental setup, observations, and key findings; and Section 5 (Conclusion) presents the conclusion and future work.

## 2. Related Works

Deep learning networks (DNNs) play a vital role in the medical field due to their significant performance in image classification when compared with human-level analysis. Hemdan et al. [11] presented a deep learning classification framework utilizing seven different CNN architectures wherein the intensity of the image using CXR was analyzed and classified into negative and positive cases. Apostolopoulos et al. [12] used a deep learning-based mobile net framework with 3905 X-ray images to develop a highly accurate approach for diagnosing pulmonary diseases. Although COVID-19 cases were classified using pretrained models, this pretrained model caused an unbalanced dataset effect on training. Litjens et al. [13] studied and analyzed various research papers on deep learning algorithms, out of which image classification, object detection, segmentation, registration, and other deep learning methods have survived.

Afshar et al. [14] proposed an alternative modeling framework named capsule network (CAPS) to handle a small dataset that performed better than the CNN-based model; its architecture was composed of several capsules with a small number of trainable parameters and convolution layers. Waheed et al. [15] developed an auxiliary classifier generative adversarial network (ACGAN) to produce CXR images. However, due to the COVID-19 outbreaks, gathering a significant number of CXR images within a short period has been challenging. The CovidGAN image generated for COVID-19 detection can be used to improve CNN performance.

Bellemo et al. [16] proposed a GAN-based classifier to develop retinal fundus images that are compatible with synthetic databases.

Xie et al. [17] examined RT-PCR outcomes in five patients with unfavorable results. The doctor conducted regular swab examinations for all patients and was finally diagnosed with COVID-19.

Du et al. [18] identified COVID-19 clinical features in children and adults. They investigated 67 cases involving 53 adults and 14 children from two research centers. The results indicated significant lung injuries in children.

Wang et al. [2] developed a COVID-19 detection method using CXR images and introduced an open COVID-Net benchmark dataset consisting of 13,975 CXR images from 13,870 patients.

Alyasseri et al. [19] reviewed comprehensive work on COVID-19 using deep learning and machine learning. They summarized previous studies on COVID-19 and concluded that CNN primarily uses a deep learning algorithm.

Al-Waisy et al. [20] proposed a method to diagnose COVID-19 using chest radiography images. It is represented as a COVID-DeepNet system that eliminates noise and enhances the contrast of the CXR images through contrast-limited adaptive histogram equalization (CLAHE) and Butterworth bandpass filter. A large dataset named COVID19-vs was created for evaluating the COVID-DeepNet system. However, the primary limitation of this method is that it can only classify the input images into healthy and COVID-19 infected.

Abed et al. [21] proposed an approach to identify COVID-19 diseases that discriminates between healthy and COVID-19 cases using traditional learning methods such as ANN, SVM, linear kernel and radial basis function, decision tree, *k*-nearest neighbor, and deep learning pretrained models using the large X-ray dataset [22] for training and testing the models.

Mohammed et al. [23] evaluated and benchmarked the scientific literature on COVID-19 diagnosis models. Multicriteria decision-making (MCDM) is integrated with TOPSIS and is ranked as the best diagnostic method based on measured criteria. According to the MCDM and TOPSIS analysis, SVM linear attains the first rank whereas SVM polynomial attains the worst rank.

Inspired by numerous research works, Agrawal et al. [24] designed an automatic method for COVID-19 detection wherein COVID-Net was pretrained on the ImageNet dataset. The architecture of COVID-Net was compared with the architectures of VGG-19 and ResNet-50 to evaluate the positive predictive value. The medical dataset can be publicly accessible under specific conditions. To train our model, we needed a large COVID-19 dataset, which is a challenging task. At the same time, the limited dataset could collapse due to the blurring and repetition of images. To resolve this, we suggested an extension of synthetic data, such as DCGAN as it can incorporate high-frequency information and features from the input data where traditional methods are not accessible. Therefore, DCGAN was used with more vital features to transfer learning extracts and was applied to a discriminator that could discriminate between CXR images. Therefore, the discriminator learned to differentiate the actual CXR images and synthetically generated images that enhanced the ability of the generator to learn about the actual CXR image. Although extensive research and studies are being conducted to diagnose COVID-19, there are still issues with small datasets and inefficient results. This study is aimed at assisting medical organizations in effectively evaluating COVID-19 cases.

## 3. Proposed Method

The main objective of our proposed method is to use the DCGAN-CNN method for efficient classification of CXR images into three categories: normal, pneumonia, and COVID-19. A flow diagram of the proposed DCGAN-CNN model is depicted in Figure 2.

### 3.1. Principle of DCGAN

The proposed DCGAN is described in detail in this section. We first analyze the fundamentals of DCGAN (Section 3.1.1), followed by CNN (Section 3.1.2), and conclude with architecture of the proposed model (Section 3.1.3).

#### 3.1.1. Fundamentals of DCGAN

A generative adversarial network or GAN is an architecture of the neural network for generative modeling that has been applied in various fields, including computer vision, medical imaging, and style transfer. The fundamental aspects of GAN are based on a min–max game, often called as a zero-sum game [25].

The players of this game belong to various GAN networks called discriminators and generators. The primary objective of the discriminator is to determine whether a given sample is part of the synthetic or actual distribution. It calculates samples according to the probability value. If the probability value is close to 0.5, the discriminator produces an optimal solution that cannot distinguish between synthetic and real samples. If the probability exceeds 0.5, it means it is the actual sample. GAN is designed as an unsupervised machine learning that learns the distribution of data classes. It has better data distribution modeling and can train any generator network where CNN is used as the generator. In this model, we used 100 × 1 noise vectors that were denoted as *z*. The network started from a layer of 1024 × 4 × 4 and reached the output with a layer of 64 × 64. Thereafter, the output image was resized to specific sizes that support the evaluation models (proposed CNN, AlexNet, and GoogLeNet) for classification purposes. The discriminator processed the real CXR image to train the data and extract its features. The generated synthetic image was transferred to the discriminator network for training along with the actual CXR images. Once the discriminator extracted the valuable features in the final layer, it was transferred to CNN for classification. The general architecture of DCGAN is illustrated in Figure 3. The two neural networks, discriminator (*D*) and generator (*G*), which train this generative model are explained below.

1. A generator (*G*) is a network that uses random noise *Z* to generate images. The input data for the generator is Gaussian noise, which is a random point in the latent space
2. The discriminator (*D*) determines whether the given image is a real or synthetic distribution. It receives the input image *x* and yields the output as *D*(*x*). The generation of the output is based on the probability of *x* being a part of the real distribution. If the output of the discriminator is 1, the image determined is real; else, it is determined as synthetic

The min–max equation of adversarial network is represented in

(1) $$\begin{array}{c} \begin{array}{c} \mathrm{Min}\\ G \end{array}\begin{array}{c} \mathrm{Max}\\ D \end{array}V\left(D,G\right)=E_{x\sim p_{\text{data}}\left(x\right)}\left[\log D\left(x\right)\right]+E_{z\sim p_{z}\left(z\right)}\left[\log\left(1-D\left(G\left(z\right)\right)\right)\right]. \end{array}$$

*D* is calculated based on the log function, where *D*(*x*) = 1 is real. Based on the min–max game theory, the data are maximized or minimized by the discriminator *D*(*G*(*z*)).Thereafter, a more complex deep convolutional GAN (DCGAN) network is updated to improve the GAN performance. After 50 epochs, they resemble the original image, and the generator creates noisy images during the initial training progress.

#### 3.1.2. CNNs

CNNs are a feed-forward neural network that transfers the data in one direction and consist of convolution layers, pooling layers, and fully connected layers. In CNN, the input images are processed as a tensor, where the data are stored in an array format. The proposed CNN model was constructed with numerous hidden layers that transfer low-level features to attain high-level feature representations of data. There were four blocks of layers with two convolution layers, a max-pooling layer, and a dropout layer. The fully connected layer output was provided to the softmax layer, wherein the classification took place.

#### 3.1.3. Architecture of the Proposed Method

A deep learning algorithm typically suffers from an overfitting problem when it is trained using a small dataset. Our proposed method provides an optimum solution to resolve this drawback, thereby improving the efficiency of CXR image classification. A block diagram of the proposed method is illustrated in Figure 4. DCGAN is a multiple neural network that utilizes random noise for fake image generation by extracting the features of an input image. In the first few layers, it first extracts the local features. Thereafter, using these local features, it extracts the global features.

Until the bottleneck, the encoder and decoder, respectively, downsample and upsample the given data. In the first four layers of the generator, the input is downsampled and then the features are learned, whereas after the fifth layer, upsampling takes place to reconstruct the image. Thereafter, the discriminator classifies the generated image into real or synthetic images. The generated dataset is then provided as the input for the CNN classification process.

The proposed CNN consists of eight convolution layers, four pooling layers, four dropout layers, two flattened layers, and two fully connected layers, as presented in Table 2. In CNN, the convolution layer maps the features from the previous layer with the feature map by detecting the local conjunction. At the end of the convolution layer, the images are split into perceptrons and compressed into the feature maps. Each layer consists of several filters; the depth feature maps are estimated based on the filter count. Each filter detects a particular feature from the input image. An overview of the architecture of the DCGAN-CNN model is presented in Figure 5. The convolution layers of the proposed CNN obtain the input images as a matrix and convolve each pixel with a filter (3 × 3). Thereafter, the horizontal stride is taken over to calculate the feature map of the images.

In the pooling layer, the matrix size is reduced and the maximum value is determined. A dropout layer that updates the hidden layers based on the training phase is added to overcome the overfitting problem. In the flattening process, the feature map is converted into a one-dimensional array for transferring it to the fully connected layer. Finally, the fully connected layers classify the labels into normal, pneumonia, and COVID-19.

The aforementioned algorithm is a constituent of two iterations and was utilized for training the proposed model. Real CXR images were taken as input (x), and the output (y) was the predicted label (normal, pneumonia, and COVID-19). In the preprocessing phase, the input image (x) dimension was converted to 256 × 256. In the training phase, the samples were trained to update the weight of the model in minibatches, known as an epoch, to train the data per cycle. Noise samples were used to generate synthetic images. Using transfer models, the images were assigned in ascending order through a stochastic gradient. After the synthetic/fake image was generated, these images were assigned in descending order through the stochastic gradient. In the testing phase, the proposed CNN predicted the output label (y). In the DCGAN, many hidden layers processed each data and extracted the vital features from it. Initially, a batch of random points was chosen from the noise or latent space that supports the model to be generated. The generated samples were referred to as synthetic samples. Subsequently, the discriminator selected a batch sample based on its weight. The layers of the discriminator continually processed until the expected value was obtained. Finally, the discriminator classified the sample as an actual or synthetic image.

### 3.2. Datasets

We utilized several datasets in this study from various resources. These datasets include the COVID-19 Radiography database, the COVID Chest X-ray dataset, the COVID-19 X-ray dataset, and the CoronaHack-Chest X-Ray dataset. The COVID-19 Radiography database [26] is the winner of the Kaggle community for the COVID-19 dataset. This dataset was developed by Qatar University researchers who collaborated with clinical experts and created a chest X-ray image for COVID-19. These datasets consist of 1341 normal, 1345 viral pneumonia, and 1143 healthy images of COVID-19. The COVID Chest X-ray dataset [27] is a public dataset of chest X-rays and CT images of patients. The COVID-19 X-ray dataset [22] was developed by a Chinese team to study the chest CT image anomalies. The CoronaHack-Chest X-Ray dataset [28] was prepared to identify the X-ray images.

### 3.3. Evaluation

We utilized the MATLAB 2020a version to run the proposed CNN with an Intel i7 processor and GPU. The proposed CNN model was executed with four different datasets, wherein the input images were resized to 256 × 256. Thereafter, the mean accuracy and standard deviations of AlexNet and GoogLeNet were compared with the proposed CNN method. Lastly, the epoch values were fine-tuned to improve the accuracy of the proposed model.

## 4. Results and Discussion

To evaluate the proposed DCGAN-CNN model quantitatively, we compared it with the existing pretraining deep learning models (AlexNet, GoogLeNet). These three models were evaluated by computing four quantitative measures: accuracy, precision, recall, and area under the curve (AUC). Compared to other performance metrics, accuracy, precision, and recall provide sufficient information to validate the deep learning model effectively:

(2) $$\begin{array}{c} \text{Accuracy}=\frac{\text{TP}+\text{TN}}{\text{TP}+\text{FP}+\text{FN}+\text{TN}}, \end{array}$$

(3) $$\begin{array}{c} \text{Precision}=\frac{\text{TP}}{\text{TP}+\text{FP}}, \end{array}$$

(4) $$\begin{array}{c} \text{Recall}=\frac{\text{TP}}{\text{TP}+\text{FN}}. \end{array}$$

In Equations (2), (3), and (4), true positive (TP) and true negative (TN) represent the correctly labeled class, whereas false negative (FN) and false positive (FP) represent the misclassified labeled class. If the false negative and false positive values of the data are the same, the accuracy is high. Precision is a metric that measures the number of false positives and represents the total amount of actual positive data available. If the precision is high, the model accuracy will be high as well. To determine the negative prediction, recall assessed the false negative values in the data. We utilized four different datasets to measure the efficiency of the proposed DCGAN-CNN model with a pretrained model.

The training and testing accuracies of the models are listed in Table 3. As per the table, the COVID-19 Radiography dataset provided an efficient accuracy (98.4%) in COVID-19 detection when compared with other datasets.

In Table 4, the accuracy of each class (normal, pneumonia, and COVID-19) was evaluated for different datasets with the existing models. The CoronaHack-Chest X-Ray predicted the classes with higher accuracy (COVID-19: 98.6%, pneumonia: 97.6%, and normal: 98.8%) than other datasets.

The time elapsed for the pretrained models and the proposed model was calculated as well; the proposed CNN model provided the best computational time. The individual accuracy and the precision and recall for each class (normal, pneumonia, and COVID-19) were calculated and tabulated in Tables 4 and 5, respectively. The AUC values of the pretrained and proposed CNN models are listed in Table 6.  Table 7 compares the accuracy of the proposed DCGAN-CNN model with the existing models [21, 23]; the accuracy of the proposed model (98.6%) was higher. Figures 6–8, respectively, display the receiver operating characteristic (ROC) curves for the proposed model, GoogLeNet, and AlexNet. According to the figures, the proposed CNN model was more efficient in detecting COVID-19 from four different datasets than the pretrained models. However, although the proposed DCGAN-CNN provided a significant advantage over COVID-19 detection, it contained some shortcomings with respect to multilabel classification, time consumption, and efficiency. DCGAN-CNN could only classify three classes, thereby limiting the CXR image features.

## 5. Conclusion

This study proposed a DCGAN-based CNN model that generates synthetic CXR images using different datasets as references, thereby improving the performance of the proposed CNN for COVID-19 detection. After numerous studies, we found that the average CNN classification performance is less in COVID-19 detection with small and large publicly available datasets. The proposed CNN model with DCGAN consists of eight convolution layers with several filters, max-pooling, and drop-out layer and provides a promising solution for detecting COVID-19 images accurately. Implementing the proposed model increased the accuracy, recall, and precision of individual classes (normal, pneumonia, and COVID-19) in all the datasets. In addition, comparing the performance metric of the proposed CNN with existing pretrained models confirmed that the efficiency of the proposed model is higher than that of the other models. Our findings confirm that the proposed DCGAN-CNN has a powerful visualization and high learning ability that helps detect the different classes of normal, pneumonia, and COVID-19 robustly. We hope that our approach will be highly supportive and reliable for medical expertise. Since the current proposed method contains some shortcomings with respect to multilabel classification, time consumption, and efficiency, in the future, we will include an additional layer for CNN that will predict multilabel classes. In addition, we will improvise the DCGAN layers to enlarge the dataset for accurate prediction.

## Figures and Tables

**Figure 1:** (a) CXR image; (b) CT image.

**Figure 2:** Flow chart of the proposed DCGAN-CNN model.

**Figure 3:** General architecture of DCGAN.

**Figure 4:** Block diagram of proposed method.

**Figure 5:** Architecture of proposed CNN+DCGAN model.

**Figure 6:** Receiver operating characteristic (ROC) curve of the proposed DCGAN-CNN.

**Figure 7:** ROC curve of GoogLeNet.

**Figure 8:** ROC curve of AlexNet.

**Algorithm 1:** Proposed method.

**Table 1:** Comparative analysis between CXR and CT imaging.

CXR imaging	CT imaging
CXR visualization for medical treatment is relatively simpler.	CT scans require more space to diagnose the patients.
It provides 2D images.	It provides 3D images.
CXR is a cost-effective and straightforward method for chest imaging.	CT imaging is costly and time-consuming.
Patients are exposed to less radiation during treatment.	Patients are exposed to high radiation during treatment.
It has high sensitivity.	It has low sensitivity.
CXR imaging equipment can be cleaned easily. In addition, it has high availability.	CT imaging equipment has a complex cleaning process. In addition, it has low availability.
Portable CXR are available for diagnosing lung anomalies	Presently, portable CT scans are unavailable.
It has low risk of cross-infection.	Cross-infection is possible due to the immediate environment.

**Table 2:** Description of layers of the proposed method.

Layer's name	Type/stride	Filter
Input	Image input	—
C1	Convolution	3 × 3 Conv 32
C2	Convolution	3 × 3 Conv 32
P1	MaxPool	—
D1	Dropout	—
C3	Convolution	3 × 3 Conv 32
C4	Convolution	3 × 3 Conv 32
P2	MaxPool	—
D2	Dropout	—
C5	Convolution	3 × 3 Conv 64
C6	Convolution	3 × 3 Conv 64
P3	MaxPool	—
D3	Dropout	—
C7	Convolution	3 × 3 Conv 64
C8	Convolution	3 × 3 Conv 64
P4	MaxPool	—
D4	Dropout	—
FC1	Fully connected	256 × 9216
F1	Flatten	—
FC2	Fully connected	3 × 256

**Table 3:** Summary of results.

Dataset	Number of images	Model	Training accuracy	Testing accuracy	Time elapsed (min)
COVID-19 X-ray	188	AlexNet	90.2	92.2	24
		GoogLeNet	89.4	91.4	35
		Proposed DCGAN-CNN	93.8	94.8	30

COVID Chest X-ray	803	AlexNet	92.5	93.5	129
		GoogLeNet	88.5	90.5	135
		Proposed DCGAN-CNN	94.6	96.6	125

COVID-19 Radiography	5910	AlexNet	96.3	96.7	2563
		GoogLeNet	94.5	95.5	2660
		Proposed DCGAN-CNN	98.4	98.5	1960

CoronaHack-Chest X-Ray	5911	AlexNet	96.2	97.2	2663
		GoogLeNet	95.4	96.4	2726
		Proposed DCGAN-CNN	97.6	98.6	2116

**Table 4:** Accuracy per class.

Dataset	Model	Normal		Pneumonia		COVID-19	
		Train	Test	Train	Test	Train	Test
COVID-19 X-ray	AlexNet	90.2	89.5	89.2	88.5	90.6	91.8
	GoogLeNet	90.1	89.8	90.3	91.5	91.3	92.5
	Proposed DCGAN-CNN	92.9	91.6	93.4	91.9	95.6	94.3

COVID Chest X-ray	AlexNet	91.6	90.8	87.6	90.8	92.3	93.6
	GoogLeNet	90.5	89.5	89.5	88.5	92.2	91.1
	Proposed DCGAN-CNN	93.6	92.4	94.6	93.4	93.5	94.3

COVID-19 Radiography	AlexNet	95.6	94.8	93.6	94.3	94.5	94.9
	GoogLeNet	94.5	93.8	92.5	91.8	91.4	91.6
	Proposed DCGAN-CNN	98.2	97.9	97.4	98.2	95.7	96.8

CoronaHack-Chest X-Ray	AlexNet	96.7	95.3	90.7	90.3	95.6	96.2
	GoogLeNet	95.5	94.8	92.5	93.8	93.8	94.2
	Proposed DCGAN-CNN	98.8	98.7	98.4	97.6	98.2	98.6

**Table 5:** Recall and precision per class.

Dataset	Model	Normal		Pneumonia		COVID-19	
		Recall	Precision	Recall	Precision	Recall	Precision
COVID-19 X-ray	AlexNet	0.90	0.89	0.85	0.88	0.90	0.91
	GoogLeNet	0.91	0.90	0.86	0.89	0.87	0.88
	Proposed DCGAN-CNN	0.92	0.93	0.93	0.89	0.95	0.92

COVID Chest X-ray	AlexNet	0.91	0.88	0.84	0.87	0.89	0.90
	GoogLeNet	0.90	0.86	0.89	0.86	0.92	0.91
	Proposed DCGAN-CNN	0.93	0.92	0.94	0.91	0.92	0.94

COVID-19 Radiography	AlexNet	0.94	0.90	0.92	0.90	0.93	0.94
	GoogLeNet	0.93	0.91	0.92	0.93	0.89	0.91
	Proposed DCGAN-CNN	0.96	0.95	0.94	0.94	0.95	0.96

CoronaHack-Chest X-Ray	AlexNet	0.95	0.91	0.92	0.88	0.93	0.94
	GoogLeNet	0.92	0.90	0.91	0.92	0.91	0.92
	Proposed DCGAN-CNN	0.97	0.96	0.95	0.96	0.97	0.98

**Table 6:** Area under curve.

Dataset	GoogLeNet	AlexNet	Proposed DCGAN-CNN
COVID-19 X-ray	0.65	0.69	0.94
COVID Chest X-ray	0.71	0.76	0.96
COVID-19 Radiography	0.92	0.94	0.95
CoronaHack-Chest X-Ray	0.93	0.96	0.98

**Table 7:** Comparing the existing methods [21, 23] with the proposed DCGAN-CNN in terms of accuracy.

Sr. No.	Method	Accuracy (%)
1	Comprehensive investigation of machine learning feature extraction and classification methods [21]	94
2	Multicriteria decision-making (MCDM) method [23]	98.3
3	Proposed DCGAN-CNN method	98.6

## Data Availability

The datasets used in this research work are available at various repositories such as the Kaggle COVID-19 Radiography database, GitHub COVID Chest X-ray dataset, Kaggle COVID-19 X-ray dataset with COVID-19 CNN Pneumonia Detector, and Kaggle CoronaHack-Chest X-Ray dataset.

## Abbreviations

*G*: Generator
*D*: Discriminator
*p*_data_(*x*): Real data distribution
*X*: Sample from *p*_data_(*x*)
*Z*: Sample from *p*_*z*_(*z*)
*D*(*x*): Discriminator network
*G*(*z*): Generator network
*p*_*z*_: Generator distribution
*E*_*z*_: Encoder of generator.
